The article "Ant Colony Algorithm-Based Audit Supervision to Promote the Optimization of New Infrastructure Investment Environment" was retracted in 2023. Reasons: unreliable results or conclusions; concerns about the data; concerns about the peer review; concerns about the citations.

# Ant Colony Algorithm-Based Audit Supervision to Promote the Optimization of New Infrastructure Investment Environment

**DOI:** 10.1155/2022/7454982

**Published:** 2022-05-28

**Authors:** Feng Yuan

**Affiliations:** School of Economics and Management, JiLin Engineering Normal University, Changchun 130052, China

## Abstract

Infrastructure investment has the characteristics of high start-up cost, high initial cost, long cycle, slow recovery, high risk, and high public welfare. Maintenance after completion requires stable financial support, maintenance costs are easily affected by government agencies, and investment efficiency is significantly reduced. This article focuses on the ant colony algorithm audit and supervision to promote the optimization of the new infrastructure investment environment and understands the relevant theories of infrastructure investment on the basis of literature data, and then, the audit supervision based on the ant colony algorithm promotes the optimization of the new infrastructure investment environment. The model is constructed, and the constructed model is tested. The test results show that, first, there is a dynamic equilibrium relationship between total infrastructure investment and GDP, even if it cannot explain the potential relationship between the two. In essence, infrastructure investment has a positive impact on economic growth. As the economic level increases, the demand for infrastructure will increase and infrastructure investment will inevitably increase. Second, the level values of the first order are all nonstationary sequences; after the difference, they are all stable and have the same single integral order. The model meets the preconditions of the cointegration test.

## 1. Introduction

Major infrastructure construction projects (hereinafter referred to as large-scale projects) include infrastructure, transportation, energy, and other social and national economic projects, which are an important part of the social and national economic development [1, 2]. Especially in China, many large-scale projects have been created to ensure the stable and rapid development of the social and national economy, such as “four trillion economic development projects” and water conservancy reform projects [3, 4]. At the same time, the construction of large-scale projects often has a serious impact on the environment, and the environmental protection activities of project developers also have a significant impact on the surrounding environment [5, 6]. Therefore, environmental issues are regarded as the most critical and restrictive content of the entire project construction goal. Only when environmental protection supervision is strengthened from the beginning to the end can the project construction effectively withstand the environmental test [7, 8]. As the foundation and necessary condition of economic and social development, infrastructure can accumulate energy and add stamina for development, while lagging construction may become the bottleneck restricting development. Economic take-off is inseparable from the boost of infrastructure construction. A common experience of the rapid economic development in coastal areas and the success of some regional development is to lay a solid foundation for rapid economic growth by taking the lead in launching large-scale infrastructure construction.

The article "Ant Colony Algorithm-Based Audit Supervision to Promote the Optimization of New Infrastructure Investment Environment" was retracted in 2023. Reasons: unreliable results or conclusions; concerns about the data; concerns about the peer review; concerns about the citations.

Regarding the research on capital construction investment, some researchers believe that infrastructure construction, as the main driving force and basic force of national economic development, is one of the most basic factors for people's production and survival. Therefore, the technical level and completeness of infrastructure construction are directly related. It is related to the development trend of the national economy and the quality of people's survival, and it is regarded as one of the most important elements of national development competitiveness. In general, by strengthening investment in infrastructure and technological innovation in infrastructure, the upgrading of the industrial structure has been promoted, and a new growth point has been provided for the development of the national economy [9]. Other researchers believe that the establishment and use of infrastructure in a developing country have a very critical significance in promoting the long-term sustainable development of its economy and society. At the same time, capital construction investment not only directly promotes the development of the national economy, but also has a far greater impact on the national economy than the investment itself. Expanding construction investment can cause an exponential increase in the income level of residents and a multiplier effect of investment. Coupled with the global economic crisis and the accelerated coordination of the world's industrial economic structure, the level of progress in infrastructure construction will have a more significant impact on our country's macroeconomic structure, and this will be for Chinese companies to participate in global production and actively participate in global economic competition to overcome constraints on population issues and poverty reduction: optimizing industrial structure, reducing production costs, enhancing corporate profitability, improving the investment environment, attracting foreign investment, increasing employment opportunities, improving social welfare, and the basic subsistence security level of the people. The final result will be reflected in the GDP growth rate. Therefore, infrastructure construction has always been an issue that governments around the world are paying more and more attention to [10]. In summary, although there are more studies on capital construction investment, there are fewer studies on investment optimization. The purpose of investment optimization is to achieve the best investment effect with the same investment. Its main objectives include reasonable investment structure; the most effective use of resources; forming the largest production capacity with the fastest construction speed; promoting technological progress to the greatest extent; and maximizing the total social products and national income.

The article "Ant Colony Algorithm-Based Audit Supervision to Promote the Optimization of New Infrastructure Investment Environment" was retracted in 2023. Reasons: unreliable results or conclusions; concerns about the data; concerns about the peer review; concerns about the citations.

In this paper, the audit supervision of ant colony algorithm promotes the optimization of new infrastructure investment environment. Based on the literature data, it analyzes the status quo of our country's infrastructure investment and the characteristics and theories of large-scale infrastructure project investment decision-making and then analyzes the characteristics and theories based on ant colony algorithm. The audit supervision promotes the construction of a new infrastructure investment environment optimization model, tests the constructed model, and draws relevant conclusions through the test results.

## 2. Infrastructure Investment Research

### 2.1. The Status Quo of Our Country's Infrastructure Investment

The first mode of infrastructure investment in my country is the centralized decision-making mode, which is determined by the state and it is difficult to exert the influence of enterprises [11]. Considering the lack of funds for infrastructure construction and the financial burden of local governments trying to change infrastructure units and infrastructure construction financing mechanisms, it is necessary to gradually open the market, increase assets, release reserve purchases, and gradually introduce nonprofit organizations in the field of infrastructure investment. Although the rate of return on infrastructure investment is not high, the rate of return on cash flow is stable and the rate of return on income is low, so the innovative billing mechanism can further increase the rate of return on capital. From the perspective of decision-making process, a macroeconomic decision-making is not a scheme produced in an instant. It is a systematic project involving a large amount of economy, management, humanities, and information technology. From the proposal of problems, the formulation of plans to the evaluation, implementation, and tracking feedback of plans, there are many uncertain factors from the internal and external management system, which are more complex and difficult to grasp than ever before.

The article "Ant Colony Algorithm-Based Audit Supervision to Promote the Optimization of New Infrastructure Investment Environment" was retracted in 2023. Reasons: unreliable results or conclusions; concerns about the data; concerns about the peer review; concerns about the citations.

There are still many problems and difficulties in my country's infrastructure [12]. First, the scale of infrastructure investment is relatively insufficient. The process of urbanization is advancing rapidly, the level of infrastructure enjoyed by ordinary people has declined, and infrastructure investment is still insufficient. Second, the structure of infrastructure funds is unreasonable. The use of foreign capital, social, and public funds is relatively low, and the construction of infrastructure in many fields is monopolized by state-owned enterprises. Third, there are relatively few infrastructure financing methods. Many cities use IPOs, BOTs, TOTs, PPPs, ADRs, and ABSs and other infrastructure investment and financing processes, but the lack of financing methods and current systems and regulations has increased. Fourth, the structure of infrastructure investment is unreasonable. The structure of the infrastructure investment fund is absurd, focusing on projects, neglecting supporting facilities and rebuilding and neglecting maintenance. The regional structure of my country's infrastructure stock is unbalanced, and infrastructure investment in some states is far below the national average. In addition, due to the lagging behind construction of related systems, the imperfect government supervision and supervision system, the imperfect social credit rating system, the unclear tax reform goals, and uncertainties, the structural risks of investment still exist.

The infrastructure investment decision-making mechanism is a group decision-making process carried out by a limited number of rational decision-makers in a fuzzy and multifunctional environment. Infrastructure investment decisions are group decisions. Decision-making options have multiple characteristics. The decision-making environment is fuzzy, the decision-making behavior is bounded rationality, and the decision maker is a person with bounded rationality (see Figure 1). Infrastructure construction has the so-called “multiplier effect”; that is, it can bring total social demand and national income several times the amount of investment. Whether a country or region's infrastructure is perfect is an important foundation for its long-term, sustainable, and stable economic development.

### 2.2. Characteristics and Theories of Investment Decision-Making for Large-Scale Infrastructure Projects

#### 2.2.1. The Complexity of the Investment Decision-Making System for Large-Scale Infrastructure Projects

The decision-making process of large-scale infrastructure construction projects is a complex system, involving many interconnected and cross-related subsystems, and the relationship between the different components of each subsystem is very complicated. At the same time, because of the uncertainty and dynamics of the decision-making environment of large-scale infrastructure projects, and the long-term engineering decision-making cycle, for example, it took more than ten years from the Beijing-Shanghai high-speed rail to its completion and commissioning. From preliminary research to final approval, it is an arduous and tedious argumentation process. From the engineering perspective, the decision-making problem of major national infrastructure construction projects is itself a problem of poor structure, faced with huge ambiguities and risk factors in the decision-making process, that is, incomplete and incorrect information. A well-structured problem is often an intuitive, familiar, and easy-to-understand problem, and it is often very consistent with completely reasonable assumptions. For example, these problems are also included in the decision-making process of national key highway construction projects. Because the constructed high-speed railway system is more systematic than other transportation methods such as road transportation, the overall layout of the road network must be made at the national level in order to make a strategic, scientific, and reasonable design of the railway network. Similarly to the design of the stations along the route and the choice of routes, including a large number of demolition projects, the construction scale of the project is quite large, but it also produced a lot of funding and financial problems, and there are many coordination problems with the management project. There are different types of decision-making problems, and the usual decision-making methods are also different. Usually, procedural decisions are taken for structured issues, while nonprocedural decisions are taken for problems that constitute undesirable problems. The key step of procedural decision-making is to obtain accurate, timely, and sufficient information. Accurate information is the most basic condition of procedural decision-making. Information error is worse than no information, which makes the direction of decision-making go to the opposite. Timely information determines the timeliness of decision-making. Modern market changes thousands of times, and time is benefit. Outdated information will inevitably make decision-making passive and eventually lead to decision-making failure.

The article "Ant Colony Algorithm-Based Audit Supervision to Promote the Optimization of New Infrastructure Investment Environment" was retracted in 2023. Reasons: unreliable results or conclusions; concerns about the data; concerns about the peer review; concerns about the citations.

#### 2.2.2. The Multiagent Nature of Investment Decisions for Large Infrastructure Projects

The complexity of decision-making for large-scale infrastructure construction projects fundamentally determines that individuals cannot participate in decision-making. In investment decision-making, the coordination of the rights and interests of all parties requires concentrated wisdom and in-depth discussions. From the perspective of decision-making units, experts and scholars in the development environment, technology, market, capital, and ecological environment of the industry are required to actively participate in investment decisions, so it may be necessary to establish a project expert group to make decisions. The decision-making of large-scale infrastructure project investment decision-making group has typical characteristics.

Group decision-making also brings uncertainty to decision-making. Making the decision to invest in a large infrastructure project brings multiple benefits. When decision-making and decision-making options are selected by different decision-makers, they inevitably have specific positions and interests, subjective tendency is large, group decision-making is difficult to coordinate the interests of all parties, and decision-making power is low. In addition, the interdisciplinary nature of decision-making obscures everyone's responsibility for project decision-making. When errors occur, everyone is evading responsibility. There are very important stages in the decision-making process-feasibility demonstration. One of the objects of feasibility demonstration is the research of decision-making procedure. Whether the methods and methods used in the demonstration procedure are logical and scientific, there are two main methods of feasibility demonstration: one is functional demonstration—that is, the “black box” method is adopted, and a large number of experiments are often used to demonstrate the feasibility of decision-making in practical demonstration—the other method is structural argumentation—that is, the degree of direct argumentation is overall, and the decisive decision-making often adopts two methods to demonstrate.

#### 2.2.3. Large-Scale Infrastructure Investment Is a Multipurpose Investment Decision

For traditional financing projects or financing projects involving the public, monetary benefits are usually regarded as the ultimate goal or the main goal of the project, while other benefits are regarded as the realization of constraints or subsidiary goals. However, the target system of major infrastructure projects is rarely unified, and the main target system of large and medium-sized infrastructure projects is generally to achieve the optimization of economic, ecological, and social benefits. In these big goal systems, each big goal is composed of multiple small goals, and these small goals not only are related to each other, but also mutually restrict each other. Therefore, WBS (Target Decomposition) is generally used to subdivide the target system of large and medium-sized infrastructure into execution levels in decision-making. In this way, a multipurpose system with hierarchical structure is composed of applications, large uses, small applications, subuses, and reference levels. In decision-making, low-level goals must follow high-level goals. In this way, different levels of goals or goals at the same level are not only related to each other, but also have opportunities to compete with each other.

The article "Ant Colony Algorithm-Based Audit Supervision to Promote the Optimization of New Infrastructure Investment Environment" was retracted in 2023. Reasons: unreliable results or conclusions; concerns about the data; concerns about the peer review; concerns about the citations.

### 2.3. Application of Artificial Ant Colony Algorithm

In the process of optimizing the route problem, the artificial ant colony algorithm requires parameter preparation, ant movement between cities, local pheromone update, and global pheromone update. The process is described as follows: first, only *m* ants are placed in *n* cities according to certain rules. Secondly, the ant traverses *n* cities according to the probability of transitioning to the specified state, so the ant prefers to choose the closest city on the path with strong pheromone content. When each ant moves from a certain city to another, it will notify all the pheromone on the path according to a certain partial pheromone update rule. At the same time, pheromone evaporates continuously over time to prevent premature pheromone concentration in certain routes. Third, each Hamilton ring is the shortest path of time that an ant is looking for. When all the ants return to the original city, a Hamilton cycle is formed. By comparing the best solution of each ant, finding and recording this section of the route to *v* are done through all the cycles. When each ant has traversed all cities and reached the starting point, the solution of the optimal path will be selected as a feasible solution, and the pheromone will be updated within a certain range according to the selected feasible solution. Finally, run multiple loop iterations and record the shortest path created after each iteration until the condition to stop the iteration is met.

There are many methods of path optimization, which can be divided into two categories: exact algorithm and heuristic algorithm. Precise algorithm refers to the algorithm that can find its optimal solution, mainly including cutting plane method, branch and bound method, and dynamic programming method. Because the amount of calculation of the accurate algorithm generally increases exponentially with the increase of the problem scale, its application range is very limited in practice.

The article "Ant Colony Algorithm-Based Audit Supervision to Promote the Optimization of New Infrastructure Investment Environment" was retracted in 2023. Reasons: unreliable results or conclusions; concerns about the data; concerns about the peer review; concerns about the citations.

## 3. Audit Supervision Based on Ant Colony Algorithm Promotes the Optimization Model of New Infrastructure Investment Environment

### 3.1. Research Purpose

The level of urban public infrastructure construction directly affects the degree of urban development. Establishing a sound financing system and scientific and reasonable allocation of investment funds are inevitable requirements for promoting urban public infrastructure construction. However, in the past, the single-purpose or standard optimization model of urban infrastructure investment income optimization models was more common, but multipurpose, multistandard, or multipurpose return on investment and multistandard model optimization are rarely included. This article focuses on the application of ant colony algorithm decision-making in the optimization model of urban public infrastructure investment and discusses the public infrastructure systems of six major cities (power supply, water supply and drainage, sewage, post, and installation).

Ants find the shortest path thanks to pheromones and environment. The intelligent behavior of ants benefits from its simple behavior rules, which make them have diversity and positive feedback. When foraging, diversity makes ants not walk into a dead end and cycle indefinitely, which is an innovative ability; positive feedback keeps good information, which is a kind of learning and strengthening ability. The ingenious combination of the two makes intelligent behavior emerge.

### 3.2. The Algorithm Principle of Portfolio Optimization

#### 3.2.1. Pheromone

Similar to the Seller-Traveler problem, this article introduces pheromone as a state variable in the portfolio problem, but it is different from the pheromone in the Seller-Traveler problem. First, this article defines pheromone as a constant parameter in the portfolio problem. As the ants look for the best, the pheromone will update. The information rules are as follows:

(1) $$\begin{array}{c} \tau_{ij}\left(t+1\right)=\rho \tau_{ij}\left(t\right)+\Delta \tau_{ij}\left(t\right). \end{array}$$

Here, *τ*_*ij*_(*t*) is the stock of pheromone on the path at time *t* (initial time, that is, when *t* = 0, *τ*_*ij*_(*t*)=*τ*(0)=0.2); *τ*_*ij*_(*t*+1) is the stock of pheromone on the path at time (*t* + 1); Δ*τ*_*ij*_(*t*) is the increment of pheromone on the path at time *t*.

There are obstacles: other ants and pheromones in the environment where ants live. Pheromones include food pheromones (left by ants who find food) and nest pheromones (left by ants who find nest). Pheromones disappear at a certain rate. Ants look for food within the range of perception. If they perceive it, they will pass. Otherwise, if you go to a place with more pheromones, each ant will make mistakes with a small probability, and not all move in the direction with the most pheromones. Ants have similar rules for finding nests and only respond to nest pheromones.

(2) $$\begin{array}{c} \eta_{ij}=\left({\bar{r}}_{j}-{\bar{r}}_{i}\right)-\left(\sigma_{j}^{2}-\sigma_{j}^{2}\right)+0.1. \end{array}$$

Among them, *η*_*ij*_ is the heuristic function between portfolio investments *i* and *j*, and ${\bar{r}}_{i}$, ${\bar{r}}_{\text{j}}$ is used to indicate the heuristic degree of investors investing *i* and *j*. r represents the previous rate of return. j and *i* are added to prevent the formation of negative numbers, and 0.1 is added to make the value of the heuristic function positive.

The article "Ant Colony Algorithm-Based Audit Supervision to Promote the Optimization of New Infrastructure Investment Environment" was retracted in 2023. Reasons: unreliable results or conclusions; concerns about the data; concerns about the peer review; concerns about the citations.

According to the set movement rules, the ant moves in the direction with the most pheromones. When there is no pheromone guidance around, it will move inertia according to the original movement direction and will remember the point passed recently to prevent turning in place. When the ant has obstacles in the direction to be moved, it will randomly choose other directions. When there is pheromone guidance, it will move according to the foraging rules.

## 4. Case Analysis

### 4.1. Investment Decision Analysis

The article selects the financial data of the top ten domestic investment companies in China, such as Beijing Capital Construction Investment Company, Tianjin Urban Infrastructure Construction Investment Company, Shanghai Municipal Infrastructure Investment Development Co., Ltd., and Beijing Zhongqing Urban Construction. In order to obtain the data, this article selects the listed urban investment subsidiary Beijing China Investment (Group) Co., Ltd., to obtain the data. This article selects the listed urban investment subsidiary Beijing China Investment Jintai Co., Ltd., as the analysis object (Code: 600683), Tianjin Capital Environmental Protection Group Co., Ltd. (Code: 600874), Shanghai Urban Investment Holdings Co., Ltd. (Code: 600649), and Chongqing Development Co., Ltd. (Code: 000514). Because the investment and construction area of the four urban investment enterprises in the shortlist is quite broad, they not only invest in local construction, but also invest in construction in other provinces and cities in China. Therefore, the article will select the most representative urban public facilities and analyze the annual average level of public building construction in Beijing, Tianjin, Shanghai, and Chongqing from 2015 to 2018 and its impact on the investment of urban investment companies. For these data, a simulation program based on ant colony calculation was established, and the simulation was run on Matlab 8.0 platform. The settings of each parameter are as follows: the group size is 1000, the maximum number of iterations is 300, the learning coefficient is 1.4964, the inertia weight range is (0.8, 1.2), and the calculation results are shown in Table 1.

The article "Ant Colony Algorithm-Based Audit Supervision to Promote the Optimization of New Infrastructure Investment Environment" was retracted in 2023. Reasons: unreliable results or conclusions; concerns about the data; concerns about the peer review; concerns about the citations.

It can be seen from Figure 2 that, from 2015 to 2018, investors mainly focused on investment in Beijing, followed by Shanghai, Chongqing, and Tianjin to maximize overall returns.

### 4.2. Model Checking

#### 4.2.1. Stationarity Test

Integration testing usually needs to measure two or more variables at the same time and produce the same single integrated sequence. Therefore, the ADF test first performs a unit root test on the sequence to see if the sequence is stable, so as to judge the integer sequence of the variable. The test conclusions are given in Table 2.

It can be seen from Figure 3 that the first-order average values are all transient series, which are fixed after first-order difference, and have the same single integration order, which meets the requirements of the test.

#### 4.2.2. Comprehensive Judgment of Criteria Such As AIC and SC

From the above ADF test results, it can be known that the first-order difference (DLNY, DLNX) of the original sequence is a constant variable, and the VAR series established with fixed variables is a fixed system. First, from the comprehensive evaluation of the lag order of AIC, SC, and other standards, the lag order of the VAR model is selected as 1. The test results are shown in Table 3.

From Figure 4, it can be found that the statistics of AIC, SC, etc., from the first row to the third row are considered to be somewhat nonautocorrelated, and all sources of unit periods are different. The model is also robust, able to analyze and perform impulse response function analysis and variance analysis.

#### 4.2.3. Granger Causality Test

The cointegration test shows that there is a dynamic equilibrium relationship between total infrastructure investment and GDP, even if it cannot explain the potential relationship between the two. In essence, infrastructure investment has a positive impact on economic growth. As the economic level increases, the demand for infrastructure will increase, which will inevitably increase infrastructure investment. Granger causality test can be used to show the relationship between the two.

It can be seen from Table 4 that, in addition to the basic LNX hypothesis, there is no LNY in the second period, and the hypothesis from the third period, namely, infrastructure investment, was rejected at a significant level of 5%. Calculating GDP growth can also see the infrastructure in the investment economy; all 2--5 periods have accepted the null hypothesis that LNY is not relevant, and GDP growth has not improved infrastructure. In the future, inflationary investment should increase moderately along with infrastructure financing.

The article "Ant Colony Algorithm-Based Audit Supervision to Promote the Optimization of New Infrastructure Investment Environment" was retracted in 2023. Reasons: unreliable results or conclusions; concerns about the data; concerns about the peer review; concerns about the citations.

## 5. Conclusions

In this paper, the audit supervision of ant colony algorithm has promoted the optimization of the new infrastructure investment environment. After analyzing the relevant theories, the audit supervision based on the ant colony algorithm has promoted the construction of a new infrastructure investment environment optimization model. The case analysis was carried out, and the model was tested. According to the experimental conclusions, the statistics from the first row to the third row of AIC, SC, etc. are considered to be somewhat nonautocorrelated, and all sources of unit cycles are different. The model is also very robust, able to analyze and perform impulse response function analysis and variance analysis.

## Figures and Tables

**Figure 1:** Infrastructure investment decision-making mechanism.

**Figure 2:** Investment decision analysis results.

**Figure 3:** Stationarity test result.

**Figure 4:** Comprehensive judgment results of AIC and SC criteria.

**Table 1:** Investment decision analysis results.

	600683	600874	600649
*t* = 1	0.29	0.25	0.25
*t* = 2	0.30	0.26	0.24
*t* = 3	0.32	0.25	0.24
*t* = 4	0.34	0.19	0.29
*t* = 5	0.36	0.17	0.29
*t* = 6	0.38	0.16	0.19
*t* = 7	0.65	0.06	0.18

**Table 2:** Stationarity test result.

	1% level	5% level	10% level
LNX	−3.73	−2.99	−2.64
DLNX	−4.34	−3.59	−3.23
LNY	−3.69	−2.98	−2.63
DLNY	−4.34	−3.59	−3.23

**Table 3:** Comprehensive judgment results of AIC and SC criteria.

	AIC	SC	HQ
0	−4.87	4.77	−4.85
1	−5.02	−4.73	−4.95
2	−4.86	−4.37	−4.73
3	−4.71	−4.02	−4.52

**Table 4:** Granger causality test.

Lag period	F-statistic	*P* value
2	2.58	0.099
	1.15	0.337

3	0.44	0.728
	3.44	0.038

4	0.45	0.773
	4.03	0.019

5	0.84	0.549
	4.12	0.019

## Data Availability

The experimental data used to support the findings of this study are available from the author upon request.
